# Pretreatment neutrophil-to-lymphocyte ratio predicts the prognosis in patients with metastatic prostate cancer

**DOI:** 10.1186/s12885-016-2134-3

**Published:** 2016-02-16

**Authors:** Takashi Kawahara, Yumiko Yokomizo, Yusuke Ito, Hiroki Ito, Hitoshi Ishiguro, Jun-ichi Teranishi, Kazuhide Makiyama, Yasuhide Miyoshi, Hiroshi Miyamoto, Masahiro Yao, Hiroji Uemura

**Affiliations:** Department of Urology, Yokohama City University, Graduate School of Medicine, Yokohama, Japan; Departments of Urology and Renal Transplantation, Yokohama City Medical Center, Yokohama, Japan; Photocatalyst Group, Special Research Laboratory, Kanagawa Academy of Science and Technology, Kawasaki, Japan; Departments of Pathology and Urology, Johns Hopkins University School of Medicine, Baltimore, USA

**Keywords:** Prostate cancer, Biomarker, Neutrophil-to-lymphocyte ratio, Metastasis

## Abstract

**Background:**

The neutrophil-to-lymphocyte ratio (NLR), a simple marker of the systemic inflammatory response in critical care patients, has been suggested as an independent prognostic factor for several solid malignancies. We investigated the utility of pretreatment NLR as a prognosticator in patients who presented with metastatic prostate cancer.

**Methods:**

We first investigated the correlation between NLR and prostate-specific antigen (PSA) levels in 1464 men who had both tests and were found to have prostate cancer on their biopsies at our institution from 1999 to 2015. We then assessed the relationship between pretreatment NLR and the prognosis in 48 patients who were diagnosed with prostate cancer metastasized to the lymph node and/or bone.

**Results:**

The NLR value was significantly elevated in men with higher PSA than in those with lower PSA (*p* < 0.001). In patients with metastatic prostate cancer, NLR (cut-off point of 3.37 determined by the AUROC curve) was correlated with both cancer-specific (*p* = 0.018) and overall (*p* = 0.008) survivals.

**Conclusions:**

Pretreatment NLR may function as a new biomarker that precisely predicts the prognosis in patients with metastatic prostate cancer.

## Background

Prostate cancer is the most common malignancy in men. The PSA screening test is widely available in Japan, but a large number of patients still present with advanced stage prostate cancer. Although most of prostate cancers with metastatic lesions respond to initial androgen ablation therapy, responders ultimately develop progressive disease of hormone refractory cancer.

The neutrophil-to-lymphocyte ratio (NLR) has been suggested as a simple marker of the systemic inflammatory response in critical care patients [1]. It has also been reported as an independent prognostic factor for several solid malignancies [2–11]. Importantly, NLR can easily be calculated from routine complete blood counts (CBCs) in peripheral blood samples [9, 10].

The utility of NLR as a potential biomarker for prostate cancer has been investigated [12]. However, most of these have included patients with advanced tumor, such as castration-resistant prostate cancer, or those who received second-line chemotherapy. To our knowledge, no studies have assessed pretreatment NLR as a predictive marker of survival in patients who were diagnosed with metastatic prostate cancer.

## Methods

### Patients and clinical and laboratory assessments

A total of 73,637 CBCs examinations that included absolute neutrophil and lymphocyte counts were performed in 9782 men at the Department of Urology, Yokohama City University Hospital (Yokohama, Japan) from 1999 to 2015. Both CBCs and PSA levels were examined in 1464 patients who were diagnosed with prostate cancer, including 48 presented with prostate cancer metastasized to the lymph node and/or bone. As the initial treatment, 42 (87.5 %) received combine androgen blockade, 8 (18.8 %) received zoledronic acid, 3 (7.1 %) underwent radical prostatectomy, and none of the patients received radiation therapy. All patients had no systemic inflammation at the time of biopsy. This study was approved by the Institutional Review Board of the Yokohama City University Medical Center. Written informed consent was obtained from all patients.

### Statistical analysis

The patients’ characteristics were analyzed using the Mann–Whitney *U*, chi-square, and one factor ANOVA tests. Any correlations between the variables were determined by the Spearman correlation analysis. The NLR cut-off value was evaluated by the AUROC curve. The Kaplan-Meier product limit estimator was used to estimate cancer-specific survival (CSS) and overall survival (OS). Survival duration was defined as the time between the dates of pathological diagnosis and death. A log-rank test was performed for comparison. The statistical analyses were performed using the Graph Pad Prism software program (Graph Pad Software, La Jolla, CA, USA). Statistical significance was determined as *p* < 0.05.

## Results

### NLR is positively associated with PSA

A total of 1464 patients with prostate cancer were analyzed in this study. Their background information, including age, white blood cell count (/mL), neutrophil (%), lymphocyte (%), and NLR are described in Tables 1 and 2. In patients with PSA of <4 ng/mL, the mean NLR was 2.57, which was increased up to 6.43 in those with PSA of ≥500 ng/mL (Fig. 1). Therefore, the NLR values were significantly higher in the high PSA level groups (*p* < 0.001). On the other hand, because of the exponential increases in the PSA levels, the correlation coefficient was not significantly different (*r* = 0.09, *p* = 0.08).

**Table 1:** Characteristics of 1464 patients with prostate cancer

Variables	*n* (%), or median (range, mean ± SD)
PSA <4	
Number of patients	738 (50.4 %)
Age (y)	76 (35–99, 75.3 ± 9.0)
WBC (/mL)	5800 (2000–16,100, 6321.3 ± 2203.3)
Neutrophil (%)	58.8 (4.5–89.0, 59.5 ± 10.3)
Lymphocyte (%)	29.0 (1.0–60.5, 28.6 ± 8.9)
NLR	2.02 (0.09–44.5, 2.57 ± 2.33)
4 ≤ PSA <20	
Number of patients	519 (35.5 %)
Age (y)	73 (44–99, 72.8 ± 8.2)
WBC (/mL)	5900 (1100–22,800, 6286.1 ± 2056.8)
Neutrophil (%)	60.5 (3.0–90.0, 60.6 ± 10.4)
Lymphocyte (%)	28.6 (3.0–91.0, 28.6 ± 9.2)
NLR	2.11 (0.03–28.67, 2.57 ± 1.99)
20 ≤ PSA < 100	
Number of patients	113 (7.7 %)
Age (y)	76 (54–104, 76.2 ± 8.9)
WBC (/mL)	6000 (1400–28,500, 6379.7 ± 3919.7)
Neutrophil (%)	61.4 (7.0–96.7, 61.6 ± 13.1)
Lymphocyte (%)	27.7 (2.6–82.5, 26.9 ± 11.9)
NLR	2.21 (0.08–37.19, 3.64 ± 4.78)
100 ≤ PSA < 500	
Number of patients	53 (3.6 %)
Age (y)	77 (59–99, 78.0 ± 8.6)
WBC (/mL)	6300 (1000–26,400, 6664.2 ± 3501.1)
Neutrophil (%)	66.0 (25.5–95, 64.1 ± 15.1)
Lymphocyte (%)	22.5 (2.5–61.0, 23.3 ± 11.9)
NLR	2.83 (0.42–38.00, 4.60 ± 5.75)
500 ≤ PSA	
Number of patients	41 (2.8 %)
Age (y)	79 (60–95, 77.3 ± 9.1)
WBC (/mL)	6400 (2300–48,800, 7973.2 ± 6909.6)
Neutrophil (%)	69.0 (29.0–60.0, 67.0 ± 14.8)
Lymphocyte (%)	20.0 (1.5–58.0, 22.2 ± 13.0)
NLR	3.33 (0.50–60.00, 6.43 ± 10.49)

**Table 2:** Patients’ background

Variables	Total	Low NLR (<3.37, *n* = 36)	High NLR (≥3.37, *n* = 12)	*p* value
Age (yr)	70.5 (71.33 ± 6.92)	70 (70.7 ± 7.2)	73.5 (73.3 ± 5.9)	0.234
iPSA (ng/mL)	82.2 (605.1 ± 1446.3)	82.2 (436.2 ± 1090.7)	102.1 (1111.7 ± 2186.0)	0.322
Pathological Grade				
Gleason’s Sum ≤ 6	2 (4.2 %)	1 (2.8 %)	1 (8.3 %)	0.156
Gleason’s Sum = 7	14 (29.2 %)	13 (36.1 %)	1 (8.3 %)	
Gleason’s Sum ≥ 8	32 (66.7 %)	22 (61.1 %)	10 (83.3 %)	
Clinical T Stage				
2	6 (12.5 %)	4 (11.1 %)	2 (16.7 %)	0.501
3	27 (56.3 %)	22 (61.1 %)	5 (41.7 %)	
4	15 (31.3 %)	10 (27.8 %)	5 (41.7 %)	
Clinical N Stage				
0	21 (43.8 %)	16 (44.4 %)	5 (41.7 %)	0.867
1	27 (56.3 %)	20 (55.6 %)	7 (58.3 %)	
Clinical M Stage				
0	13 (27.1 %)	12 (33.3 %)	1 (8.3 %)	0.091
1	35 (72.9 %)	24 (66.7 %)	11 (91.7 %)	
NLR	2.49 (2.93 ± 1.66)	2.17 (2.25 ± 0.64)	4.26 (4.98 ± 2.08)	<0.001

median (mean ± SD)

**Fig. 1:** Association between NLR and PSA levels. Each NLR value represents the mean + SEM

### NLR predicts the survival of metastatic prostate cancer

CBCs were examined in 48 metastatic prostate cancer patients before undergoing prostate needle biopsy. The basic characteristics, including age, initial PSA, and Gleason score, are shown in Table 3. There were no statistically significant correlations between NLR and each of clinicopathologic feature. The median and mean (± SD) follow-up times were 61 and 55.9 (±34.0) months, respectively. Nineteen patients (39.6 %) died of prostate cancer.

**Table 3:** Characteristics of 48 patients with metastatic prostate cancer

Variables	Median (range, mean ± SD)
Age (y)	70.5 (51–88, 71.33 ± 6.92)
Initial PSA (ng/mL)	82.16 (8.2–7285, 605.06 ± 1446.25)
Pathological Grade	
Gleason Score ≤ 6	2 (4.2 %)
Gleason Score = 7	14 (29.2 %)
Gleason Score ≥ 8	32 (66.7 %)
Clinical T Stage	
2	6 (12.5 %)
3	27 (56.3 %)
4	15 (31.3 %)
Clinical N Stage	
0	21 (43.8 %)
1	27 (56.3 %)
Clinical M Stage	
0	13 (27.1 %)
1	35 (72.9 %)
NLR	2.49 (0.84–10.56, 2.93 ± 1.66)

We created an AUROC curve to determine the NLR cut-off value for predicting the prognosis. The cut-off value was determined to be 3.37 (Fig. 2). Patients with high NLR showed significantly poorer CSS (*p* = 0.018) and OS (*p* = 0.008), compared with those with low NLR (Fig. 3).

**Fig. 2:** The AUROC for the NLR (**a**: Cancer-Specific Survival, **b**: Overall Survival)

**Fig. 3:** The Association of patient outcomes with NLR (**a**: Cancer-Specific Survival, **b**: Overall Survival)

## Discussion

PSA was also found to be positively correlated with the NLR in patients with prostate cancer. McDonald et al. hypothesized that the NLR might reflect the balance between innate (neutrophils) and adaptive (lymphocytes) immune responses; its association with higher serum PSA levels might indicate impairment in the adaptive host’s ability to control inflammation [12]. The PSA level was shown to be a prognostic factor in prostate cancer patients with a PSA of >500 ng/mL, and higher PSA levels (>1000 or 5000 ng/mL) were associated with a poorer outcome [13]. Our results also support those data.

Our results showed pretreatment NLR to be a predictor of survival in patients presenting with metastatic prostate cancer. Increasing evidence shows that the presence of systemic inflammation is correlated with poorer CSS in various solid organ tumors [3, 14–19]. Moreover, nonsteroidal anti-inflammatory medications have been suggested to reduce the risk of developing prostate cancer, implying its critical correlation with inflammation [14, 15]. Markers of systemic inflammation, including the NLR, have also been associated with elevated PSA levels in men without known prostatic disease [12]. It has previously been demonstrated that the presence of an inflammatory response can be determined by not only C-reactive protein expression but also NLR elevation [1, 3, 20].

We retrospectively investigated the NLR in our clinical database. CBCs are usually determined during clinical check-ups, and thus it is possible to apply the NLR to all patients, both preoperatively and postoperatively. The NLR can be simply calculated from routine CBCs with differentials [21]. CBCs are usually examined in the clinical check-up, and NLR can be applied to virtually all patients either before or after surgery/medical treatment. The NLR that has been proposed to estimate the magnitude of systemic inflammation in cancer patients is thus an easily and inexpensively measured prognostic marker [2, 22–24].

The proposed mechanisms involving the relationship between NLR elevation and tumor progression include the increased supply of growth factors, survival factors, pro-tumorigenic factors, and extracellular matrix-modifying enzymes (which can facilitate invasion and metastasis), and inductive signals that may lead to epithelial-to-mesenchymal transition [21, 25]. Patients with an elevated NLR have also been shown to exhibit a lymphocyte-mediated immune response to malignancy, suggesting that NLR elevation could be associated with an increased potential for tumor progression and a worse prognosis [26, 27]. The interaction between the tumor and the host immune system promotes tumor cell proliferation and metastasis, and activates the inflammatory cascade in the host, which leads to the further deterioration of the general condition of cancer patients [28]. Studies have proposed that tumor-associated neutrophils have two different states: anti-tumorigenic (N1-phenotype) and a pro-tumorigenic (N2-phenotype) [29, 30]. CD8-positive lymphocytes are also known to play an anti-tumorigenic role [29, 31].

The present study is associated with some limitations due to its retrospective nature. Our patients received a variety of prostate cancer therapies including traditional hormonal treatment as well as several new drugs. Although the treatment options were heterogeneous, we found the NLR to be a new biomarker that was associated with patient outcomes. Thus, pretreatment NLR may be a useful prognosticator in patients with metastatic prostate cancer. The second one is that NLR may be affected by infection, systemic inflammation and medication, however, such conditions may not have affected the NLR in our cohort since the NLR was obtained at the time of biopsy and any cases with infection or systemic inflammation were excluded from the analysis. In addition, none of the patients received any pre-biopsy medication that is known to affect the NLR. The third limitation is the limited sample size. As a result, further study with a larger group of patients is needed.

## Conclusions

In conclusion, pretreatment NLR may function as a new biomarker that precisely predicts the prognosis in patients with metastatic prostate cancer.

### Availability of supporting data

Due to ethical restrictions, the raw data underlying this paper is available upon request to the corresponding author.

## Abbreviations

CBCs: complete blood counts
CSS: cancer-specific survival
NLR: neutrophil-to-lymphocyte ratio
OS: overall survival
PSA: prostate-specific antigen
